This article has been retracted.

# Apoptosis and Molecular Targeting Therapy in Cancer

**DOI:** 10.1155/2014/150845

**Published:** 2014-06-12

**Authors:** Mohamed Hassan, Hidemichi Watari, Ali AbuAlmaaty, Yusuke Ohba, Noriaki Sakuragi

**Affiliations:** ^1^Biotechnology Program, Department of Zoology, Port Said University, Faculty of Science, Port Said 42521, Egypt; ^2^Department of Obstetrics and Gynecology, Graduate School of Medicine, Hokkaido University, Sapporo 060-8638, Japan; ^3^Department of Cell Physiology, Graduate School of Medicine, Hokkaido University, Sapporo 060-8638, Japan

## Abstract

Apoptosis is the programmed cell death which maintains the healthy survival/death balance in metazoan cells. Defect in apoptosis can cause cancer or autoimmunity, while enhanced apoptosis may cause degenerative diseases. The apoptotic signals contribute into safeguarding the genomic integrity while defective apoptosis may promote carcinogenesis. The apoptotic signals are complicated and they are regulated at several levels. The signals of carcinogenesis modulate the central control points of the apoptotic pathways, including inhibitor of apoptosis (IAP) proteins and FLICE-inhibitory protein (c-FLIP). The tumor cells may use some of several molecular mechanisms to suppress apoptosis and acquire resistance to apoptotic agents, for example, by the expression of antiapoptotic proteins such as Bcl-2 or by the downregulation or mutation of proapoptotic proteins such as BAX. In this review, we provide the main regulatory molecules that govern the main basic mechanisms, extrinsic and intrinsic, of apoptosis in normal cells. We discuss how carcinogenesis could be developed via defective apoptotic pathways or their convergence. We listed some molecules which could be targeted to stimulate apoptosis in different cancers. Together, we briefly discuss the development of some promising cancer treatment strategies which target apoptotic inhibitors including Bcl-2 family proteins, IAPs, and c-FLIP for apoptosis induction.

## 1. Introduction

Apoptosis is a very tightly programmed cell death with distinct biochemical and genetic pathways that play a critical role in the development and homeostasis in normal tissues [1]. It contributes to elimination of unnecessary and unwanted cells to maintain the healthy balance between cell survival and cell death in metazoan [2, 3]. It is critical to animals especially long-lived mammals that must integrate multiple physiological as well as pathological death signals. Evidence indicates that insufficient apoptosis can manifest as cancer or autoimmunity, while accelerated cell death is evident in acute and chronic degenerative diseases, immunodeficiency, and infertility. Under many stressful conditions like precancerous lesions, activation of the DNA damage checkpoint pathway can serve to remove potentially harmful DNA-damaged cells via apoptosis induction to block carcinogenesis [4, 5]. Thus, the apoptotic signals help to safeguard the genomic integrity [3, 6, 7] while dysregulation of the apoptotic pathways may not only promote tumorigenesis but also render the cancer cell resistant to treatment. Thus, the evasion of apoptosis is a prominent hallmark of cancer [8]. Cancer cells are, in fact, harboring alterations that result in impaired apoptotic signaling, which facilitates tumor development and metastasis [6–8].

Here, we provide an overview of mechanisms by which the main regulatory molecules govern apoptosis in normal cells and describe models of apoptotic dysregulation based on alterations in their function that facilitate the evasion of apoptosis in cancer cells. We will also briefly discuss the development of some promising cancer treatment strategies based on targeting the apoptotic inhibitor to stimulate the apoptotic signals. We will shed some light on this very active field of endeavor that witnessed many breakthroughs over the last few years. Notably, insights from proposed target molecules have included different portions of the death pathway depending on the type of cancer. Applications of many of such targeted therapy in different cell types and signals studied in them have emphasized selected control points for each targeted therapy.

## 2. Apoptosis Defect and Cancer

Defects in programmed cell death (apoptosis) mechanisms play important roles in tumor pathogenesis, allowing neoplastic cells to survive over intended lifespans, subverting the need for exogenous survival factors and providing protection from oxidative stress and hypoxia as the tumor mass expands. That gives time for accumulation of genetic alterations that deregulate cell proliferation, interfere with differentiation, promote angiogenesis, and increase invasiveness during tumor progression [9]. Apoptosis defects are now considered an important complement of protooncogene activation, as many deregulated oncoproteins that drive cell division also trigger apoptosis (e.g., Myc, E1a, and Cyclin-D1) [10]. On the other hand, the noncancerous cells have a DNA repair machinery. Defects in DNA repair and/or chromosome segregation normally trigger cell suicide as a defense mechanism for eradicating genetically unstable cells and thus such suicide mechanism's defects permit survival of genetically unstable cells, providing opportunities for selection of progressively aggressive clones and may promote tumorigenesis [11].

There are varieties of molecular mechanisms that tumor cells use to suppress apoptosis. Tumor cells can acquire resistance to apoptosis by the expression of antiapoptotic proteins such as Bcl-2 or by the downregulation or mutation of proapoptotic proteins such as BAX. Since the expression of both Bcl-2 and BAX is regulated by the p53 tumor suppressor gene [12], some forms of human B-cell lymphoma have Bcl-2 overexpression. That example represents the first and strongest lines of evidence that failure of cell death contributes to cancer [13].

Apoptosis defects may allow epithelial cells to survive in a suspended state, without attachment to extracellular matrix which facilitate metastasis [14]. They also promote resistance to the immune system, including many weapons of cytolytic T cells (CTLs) and natural killer (NK) cells used for attacking tumors that depend on integrity of the apoptosis machinery [15]. Cancer-associated defects in apoptosis play a role in treatment resistance with conventional therapies like chemotherapy and radiotherapy, increasing the threshold for cell death and thereby requiring higher doses for tumor killing agents [16]. Thus, dysregulated or defective apoptosis regulation is a fundamental aspect of the tumor biology. Successful eradication of cancer cells by nonsurgical means is ultimately approached via induction of apoptosis. Therefore, all the cancer drug designers try either to activate the inactivated apoptotic mechanism or rectify a defective one. Hence, all cytotoxic anticancer therapies currently in clinical use, when they work, induce apoptosis of malignant cells. Hence, deeper understanding of the molecular mechanisms of apoptosis and its defective status opens the gate for a new class of targeted therapeutics.

### 2.1. Induction of Apoptosis

Apoptosis is caused by proteases, known as “caspases,” which specifically target cysteine aspartyl [17, 18]. Upon receiving specific signals instructing the cells to undergo apoptosis a number of distinctive changes occur in the cell. A family of proteins known as caspases is typically activated in the early stages of apoptosis. These proteins cleave key cellular components that are required for normal cellular function including structural proteins in the cytoskeleton and nuclear proteins such as DNA repair enzymes. The caspases can also activate other degradative enzymes such as DNases, which begin to cleave the DNA in the nucleus.

During the apoptotic process, apoptotic cells display distinctive morphology. Typically, the cell begins to shrink following the cleavage of lamins and actin filaments in the cytoskeleton. The apoptotic breakdown of chromatin in the nucleus often leads to nuclear condensation and/or a “horse-shoe” like appearance. Cells continue to shrink, packaging themselves into a form that allows for their removal by macrophages. These phagocytic cells are responsible for clearing the apoptotic cells from tissues in a clean and tidy fashion that avoids many of the problems associated with necrotic cell death. In order to promote their phagocytosis by macrophages, apoptotic cells often undergo plasma membrane changes that trigger the macrophage response. One of such changes is the translocation of phosphatidylserine from the inside of the cell to the outer surface. The end stages of apoptosis are often characterised by the appearance of membrane blebs or blisters process and small vesicles called apoptotic bodies.

The real workers in apoptosis mechanism are caspases. Caspases family is composed of intracellular cysteine proteases (*n* = 11 in humans), which collaborate in proteolytic cascades. These caspases activate themselves and each other. Within these proteolytic cascades, caspases can be positioned as either upstream “initiators” or downstream “effectors” of apoptosis. Several pathways for activating caspases exist.

First, there are thirty members of the tumor necrosis factor- (TNF-) family receptors; eight contain a so-called death domain (DD) in their cytosolic tail [19]. Several of these DD-containing TNF-family receptors use caspase activation as a signaling mechanism, including TNFR1/CD120a, Fas/APO1/CD95, DR3/Apo2/Weasle, DR4/TrailR1, DR5/TrailR2, and DR6. Ligation of these receptors at the cell surface results in the recruitment of several intracellular proteins, including certain procaspases, to the cytosolic domains of these receptors, forming a “death-inducing signaling complex” (DISC) that triggers caspase activation, constituting the so-called “extrinsic” pathway for apoptosis [20]. The caspase-8 and, in some cases, caspase-10 are the specific caspases summoned to the DISC. These caspases contain so-called death effector domains (DEDs) in their N-terminal prodomains that bind to a corresponding DED in the adaptor protein, FADD, thus linking them to the TNF-family death receptor complexes.

Second is the intrinsic pathway, in which mitochondria induces apoptosis by releasing cytochrome-c (cyt-c) into the cytosol. The released cytochrome c assembles a multiprotein caspase-activating complex, referred to as the “apoptosome” [21]. The central component of the apoptosome is Apaf1, a caspase-activating protein that oligomerizes upon binding cyt-c and then binds procaspase-9 via interaction with its caspase recruitment domain (CARD). The intrinsic pathway is activated by myriad stimuli, including growth factor deprivation, oxidants, Ca2^+^ overload, oncogene activation, DNA-damaging agents, and microtubule targeting drugs. In addition to cyt-c, mitochondria also releases endonuclease G, AIF (a death modulating flavor protein), and IAP antagonists SMAC (DIABLO) and OMI (HtrA2). Some of these molecules may promote caspase-independent (nonapoptotic) cell death [22, 23].

A third pathway for apoptosis induction is specific to CTL and NK cells, which spray apoptosis-inducing protease, granzyme B (GraB), onto target cells. GraB then piggybacks into cells via mannose-6-phosphate receptors (IGFR2) and enters effective cellular compartments via perforin channels [24]. GraB is a serine protease but, similar to the caspases, it cleaves substrates at Asp residues, including several caspases and some caspase substrates. The fourth pathway is a caspase activation pathway. This pathway is proposed to be linked to endoplasmic reticulum (ER)/Golgi stress [17]; however, many mechanistic details are lacking. Finally, a nuclear pathway for apoptosis regulation was proposed. That pathway depends on discrete nuclear organelles, called Pml oncogenic domains (PODs) or nuclear bodies (NBs). Ablation of the pml gene in mice results in general resistance to apoptosis through unknown mechanisms. Several proteins that can promote apoptosis have been localized to PODs, including Daax, Zip kinase, and Par4, and defects in assembly of these nuclear structures are documented in cancers [25]. How PODs are linked to caspase activation pathways is unknown. Several endogenous antagonists of the caspase-activation pathways have been discovered and examples of dysregulation of their expression or function in cancers have been obtained. These apoptosis mediators help cells to decide successful apoptosis or unsuccessful one. They sometimes act as targets for drug discovery, with the idea that abrogating their cytoprotective functions may restore apoptosis sensitivity to tumor cells.

### 2.2. Resistance to Apoptosis in Cancer

Cancer is an example where the normal mechanisms of cell cycle regulation are dysfunctional, with either an over-proliferation of cells and/or decreased removal of cells [26]. In fact, suppression of apoptosis during carcinogenesis is thought to play a central role in the development and progression of some cancers [27]. There is a variety of molecular mechanisms that tumor cells use to suppress apoptosis.

### 2.3. Carcinogenesis via Intrinsic Signaling Defects

Mitochondria-dependent apoptosis is one of the most important pathways for apoptosis induction. That is why disturbing this pathway is an effective way to inhibit apoptosis. Bcl-2 family proteins (*n* = 24 in humans) are central regulators of the intrinsic pathway, which either suppress or promote changes in mitochondrial membrane permeability required for release of cyt-c and other apoptogenic proteins [21, 24]. Antiapoptotic proteins (e.g., Bcl-2, Bcl-xL, Bcl-W, Mcl-1, and Bfl-1/A1), which display sequence homology in all BH1-BH4 domains, promote cell survival, whereas proapoptotic proteins mediate receptor-, mitochondria-, or endoplasmic reticulum (ER) stress-dependent apoptosis. The latter group is subdivided into multidomain or BH3-only proteins. The former consists of Bax and Bak, which are essential for apoptosis [28]. The BH3-only proteins are further divided into two subclasses: “activators” (e.g., Bim and tBid), which directly activate Bax/Bak to induce mitochondrial outer membrane permeabilization (MOMP), and “sensitizers/derepressors” (e.g., Bad, Bik, Bmf, Hrk, Noxa, and Puma), which do not activate Bax/Bak directly but instead neutralize antiapoptotic proteins [29, 30]. The central role that Bax/Bak play in apoptosis is supported by evidence that BH3-only proteins fail to trigger apoptosis in Bax/Bak-deficient cells [31, 32]. Antiapoptotic proteins block death signaling by antagonizing the actions of Bax/Bak through partially known mechanisms. As recently summarized, antiapoptotic proteins prevent Bax/Bak activation by sequestering/inhibiting “activator” BH3-only proteins and/or directly inhibiting Bax/Bak activation [33]. “Sensitizer” BH3-only proteins displace “activator” BH3-only proteins from antiapoptotic proteins, leading to Bax/Bak activation. Alternatively, BH3-only proteins may directly neutralize/inhibit antiapoptotic proteins, releasing their inhibition of Bax/Bak.

Overexpression of antiapoptotic Bcl-2 or Bcl-xL probably occurs in more than half of all cancers [34], rendering tumor cells resistant to myriad apoptotic stimuli, including most cytotoxic anticancer drugs. For example, forced expression of Bcl-2 protein from plasmid vectors, in contrast, abrogates sensitivity to the apoptosis promoting effects of antiestrogens in breast cancer lines, while antisense Bcl-2 prevents estrogen-mediated apoptosis suppression, thus establishing a direct functional connection between ER and Bcl-2 and suppression of apoptosis [35].

### 2.4. Carcinogenesis via Extrinsic Pathway Signaling Defect

The extrinsic pathway is activated* in vivo* by TNF family ligands that engage DD-containing receptors, resulting in activation of DED-containing caspases. The “death ligands” are expressed on CTLs, NK cells, and other types of immune-relevant cells (activated monocytes/macrophages and dendritic cells) and are used as weapons for eradication of transformed cells [19]. Mice-based studies on genetic alterations in genes encoding death ligands or their receptors, as well as use of neutralizing antibodies and Fc-fusion proteins, have provided evidence of important roles in tumor suppression by cellular immune mechanisms. Fas ligand (FasL) is important for CTL-mediated killing of some tumor targets, and TRAIL (Apo2 ligand) is critical for NK-mediated tumor suppression. Some tumor cells resist the response of the death receptor pathway to FasL produced by T cells to evade immune destruction. Many tumor cell lines display intrinsic resistance to TRAIL even though they express the necessary cell surface receptors confirming that, during evolution of tumors* in vivo*, selection occurs for malignant clones capable of withstanding immune attack. This could occur in a variety of ways including downregulation of the Fas receptor, expression of nonfunctioning Fas receptor, and secretion of high levels of a soluble form of the Fas receptor. That will directly sequester the Fas ligand or expression of Fas ligand on the surface of tumor cells (reviewed, [36]). Some tumor cells are capable of a Fas ligand-mediated “counter attack” that results in apoptotic depletion of activated tumor infiltrating lymphocytes [37]. Thus, successful biological therapy depends on restoring competency of the extrinsic pathway.

Another molecule is the c-FLIP, cellular FADD-like interleukin-1beta-converting enzyme inhibitory proteins long c-FLIP(L), which regulates caspase-8 activation. Despite the identified dual functionality of c-FLIPL as a pro- or antiapoptotic factor in normal tissues, c-FLIPL has generally been shown to act as a key negative regulator of apoptosis in human cancer cells [38, 39]. Increased expression of c-FLIP has been detected in many human malignancies, including melanoma, hepatocellular carcinoma [40], nonsmall cell lung carcinoma [40], and endometrial [41], colon [42], and prostate cancer [43–45]. While its overexpression has been associated with cancer progression and/or poor prognosis in BL, HCC, and ovarian, endometrial, colon, and prostate cancer [38, 39, 42, 46], elevated expression of c-FLIP blocks caspase-8 and renders cells resistant to cell receptor-mediated apoptosis [38]. Overexpression of c-FLIP_L_ has been reported to bind proteins involved in these signaling pathways, including TRAF1, TRAF2, RIP, and RAF1, and thereby promotes the activation of NF-*κβ* and ERK as downstream molecules [39].

In TRAIL-resistant nonsmall cell lung cancer (NSCLC) cells, c-FLIP and RIP, have been shown to be essential for TRAIL-induced formation of the DISC in nonraft domains of the plasma membrane and consequent activation of NF-*κβ* and ERK cell survival signals. In contrast, knockdown of c-FLIP has been found to redistribute the DISC to lipid rafts and switch DISC signaling to TRAIL-induced apoptosis [47]. NF-*κβ* constitutive activation has been linked to the pathogenesis of many human cancers [48], and inhibition of NF-*κβ*-induced transcription of c-FLIP has been shown to sensitize cells to death receptor-mediated apoptosis [49, 50]. NF-*κβ*-mediated upregulation of c-FLIP is implicated as an important factor in the evasion of cell death by cancer cells.

### 2.5. Carcinogenesis via Convergence Pathway Inhibition

The intrinsic and extrinsic pathways for caspase activation converge on downstream effector caspases. Mechanisms for suppressing apoptosis at this distal step have been revealed, and their relevance to cancer is becoming progressively clear. In this regard, the apoptosis-inhibiting proteins (IAPs) represent a family of evolutionarily conserved apoptosis suppressors (*n* = 8 in humans), many of which function as endogenous inhibitors of caspases. All members of this family, by definition, contain at least one copy of a so-called BIR (baculovirus iap repeat) domain, a zinc binding fold, which is important for their antiapoptotic activity, present in 1–3 copies. Caspases-3 and -7, as well as caspase-9 (intrinsic pathway), are directly affected by the human IAP family members, XIAP, cIAP1, and cIAP2. For XIAP, the second BIR domain and the linker region between BIR1 and BIR2 are required for binding and suppressing caspases-3 and -7, while the third BIR domain binds caspase-9. Thus, different domains in the multi-BIR containing IAPs are responsible for suppression of different caspases. IAP family member Livin (ML-IAP) contains a single BIR and inhibits caspase-9 but not caspase-3 and -7. Survivin also contains a single BIR which associates with caspase-9.

IAPs are overexpressed in many cancers, while more detailed information is needed about the exact deregulation of the 8 members of this gene family in specific types of cancer. Those IAPs elevations found in cancers are important for maintaining tumor cell survival and resistance to chemotherapy as confirmed by antisense-mediated reductions experiments. Targeting IAP-family members XIAP, cIAP1, Survivin, or Apollon can induce apoptosis in tumor cell lines in culture or sensitize cells to cytotoxic anticancer drugs.

Endogenous antagonists of IAPs keep these apoptosis suppressors in check, promoting apoptosis. Two of these naturally occurring IAP-antagonists, SMAC (Diablo) and HtrA2 (Omi), are sequestered inside mitochondria, becoming released into the cytosol during apoptosis [51]. SMAC and HtrA2 have N-terminal leader sequences that are truncated by proteolysis upon import into mitochondria, exposing a novel tetrapeptide motif that binds the BIR domains of IAPs. These IAP antagonists compete with caspases for binding to IAPs, thus freeing caspases from the grip of the IAPs and promote apoptosis. Thus, some modern synthetic peptides-based therapeutics that mimic SMAC and HtrA2 trigger apoptosis or sensitize tumor cell lines to apoptosis induced by cytotoxic anticancer drugs or TRAIL* in vitro* and even in some tumor xenograft models [52].

### 2.6. How the Cancer Cells Overcome the Therapeutic Agents-Induced Apoptosis

The success of each therapeutic strategy depends mainly on the ability of the therapeutic tool to induce apoptosis either by targeting the overexpressed antiapoptotic proteins or by stimulating the expression of the proapoptotic molecules. However, many of the therapeutic agents are still challenged by maneuvering(s) from the cancer cells to survive treatments. Alterations in the expression levels or mutation of a chemotherapeutic drug's target(s) may have an impact on apoptosis by such drug. Here, we list some of the mechanisms by which cancer cell can overcome three of the standard therapeutic agents.

#### 2.6.1. 5-Fluorouracil (5-FU)

The fluoropyrimidine 5-fluorouracil (5-FU) is widely used in cancer treatment including colorectal and breast cancer treatments [53, 54], but resistance to that drug remains a major clinical obstacle; 5- is part of its antitumor activity and FU targets the tumor suppressor p53 and subsequently triggers the cell cycle. 5-FU-induced apoptosis is p53-dependent; however, apoptosis can also occur in p53 mutant cell lines by a mechanism still unknown [55–57]. 5-FU is an analogue of uracil with a fluorine atom at the C5 position of the pyrimidine ring. Inside cells, 5-FU is converted into different active metabolites, including fluorodeoxyuridine monophosphate (FdUMP), fluorodeoxyuridine triphosphate (FdUTP), and fluorouridine triphosphate (FUTP). These metabolites have been implicated in both global RNA metabolism due to the incorporation of the ribonucleotide FUMP into RNA and DNA metabolism due to thymidylate synthase (TS) inhibition or direct incorporation of FdUMP into DNA, leading to a wide range of biological effects which trigger apoptotic cell death. The inhibition of TS is believed to be the primary anticancer activity of 5-FU [58, 59]; however, 5-FU has been shown to acutely induce TS expression in both cell lines and tumors [60]. This induction of TS seems to be due to inhibition of a negative feedback mechanism in which ligand-free TS binds to its own mRNA and inhibits its own translation [61]. When stably bound by FdUMP, TS can no longer bind its own mRNA and suppress translation, resulting in increased protein expression. This constitutes a potentially important apoptosis resistance mechanism, as acute increases in TS would facilitate recovery of enzyme activity. Thus, TS expression acted as a key determinant of 5-FU sensitivity [62] while* in vitro* studies have validated the association between TS expression and apoptosis 5-FU [63, 64] while the improved response rates of 5-FU-based chemotherapy were observed in patients with low tumour TS expression [65, 66]. Recently, genotyping studies have found that patients homozygous for a particular polymorphism in the TS promoter (TSER3/TSER3) that increases TS expression are less likely to respond to 5-FU-based chemotherapy than patients who are heterozygous (TSER2/TSER3) or homozygous for the alternative polymorphism (TSER2/TSER2) [67]. Collectively, many evidences indicate that high TS expression correlates with increased 5-FU resistance.

#### 2.6.2. Antimicrotubule Agents (AMA)

Microtubules are highly dynamic cytoskeletal fibres composed of tubulin subunits (most commonly *α*- and *β*-tubulin) that have crucial roles in maintaining cell shape, in cell signalling, in cell division and mitosis, and in the transport of vesicles and mitochondria and other cellular components throughout the cell [68]. The rapid polymerization/depolymerization dynamics of microtubules are critical for proper spindle function and accurate chromosome segregation during mitosis.

Taxanes, such as paclitaxel and docetaxel, and vinca alkaloids, such as vinblastine and vincristine, suppress microtubule polymerization dynamics, which results in the slowing or blocking of mitosis at the metaphase-anaphase boundary [69]. These compounds can block or slow mitosis and subsequently cells eventually die by apoptosis [70]. Microtubule polymer levels and dynamics are regulated by many factors, including expression of different tubulin isotypes [71]. Cells can resist paclitaxel and vinca alkaloids by changing the microtubules dynamics and levels of tubulin isotypes [72–74]. Sometimes, a reduction in total intracellular tubulin levels could be observed in paclitaxel-resistant cells. Therefore, the development of resistance to antimicrotubule agents may involve changes in the microtubule polymer mass and expression of different tubulin isotypes. Furthermore, specific *β*-tubulin mutations that alter sensitivity to paclitaxel have been reported* in vitro *[75–77]. The clinical relevance of these mechanisms of resistance to antimicrotubule agents remains to be determined.

#### 2.6.3. Cisplatin

The therapeutic activity of cisplatin and carboplatin is mediated by an active species, formed by aqueous hydrolysis as the drug enters the cell. This active species interacts with DNA, RNA, and protein, but the cytotoxic effect seems to be primarily mediated via the formation of DNA interstrand and intrastrand crosslinks. These platinum-DNA adducts are recognized by a number of proteins, including those involved in nucleotide excision repair (NER), mismatch repair (MMR), and high-mobility group proteins (such as HMG1 and HMG2) [78]. Platinum-induced DNA damage is normally repaired by the NER pathway, whereas the MMR pathway seems to trigger apoptosis [79, 80]. The mechanism by which damage recognition results in apoptosis is unclear; however,* in vitro *data support a role for cisplatin-mediated activation of the c-ABL and JNK/SAPK pathway in apoptotic signalling in MMR-proficient cells [81]. In addition, the induction of p53, possibly by the ATM-CHK2 pathways, following DNA strand breaks leads to apoptosis via the intrinsic pathway and also contributes to the cytotoxicity of cisplatin [82].

Bcl-2 members are localized in the mitochondria and have either proapoptotic (Bax, Bak, Bid, and Bim) or antiapoptotic (Bcl-2, Bcl-xL, and Bcl-W) functions [8, 83, 84]. These members are involved in the downstream action by cisplatin. These proteins form either homodimers (such as Bcl-2/Bcl-2) or heterodimers (e.g., Bcl-2/Bax) depending on the levels present of each component. Excess level of homodimers can either inhibit (e.g., Bcl-2/Bcl-2) or induce (e.g., Bax/Bax) apoptosis. Although it is not confirmed whether cisplatin can directly modulate levels of the antiapoptotic protein or not, there is evidence that cisplatin significantly transactivates the* bax* gene by wild-type p53. Thus, an increase in the Bax to Bcl-2 ratio by cisplatin-induced p53 has been reported to activate the apoptotic process [85]. However, extrapolating experimental results to the clinic results needs much caution, for instance, the demonstration that experimental overexpression of* bcl-2 *in tumors leads to the expected cisplatin resistance [86–88]. That was opposite to a clinical study, which reported that cisplatin surprisingly improved survival of ovarian cancer patients with increased* bcl-2* gene expression [87]. Now, it is understood that proapoptotic homodimers affect cisplatin-induced apoptosis by first stimulating the mitochondria to release cytochrome* c*, which in turn activates a series of proteases that includes caspase-1, -3, and -9 [84, 89–91] which are the final effectors of drug mediated apoptosis.

## 3. Molecular Targeting Therapies and Apoptosis

Expression of inhibitors of apoptosis as well as inactivation of apoptosis promoters is observed in human cancers [92]. Moreover, functional defects in apoptotic signal transduction may translate into drug resistance of cancer [86, 93]. Over the past decade, significant advances have been made in discovery and validation of several types of novel cancer therapeutics. Such novel therapeutics tries to prime the apoptotic machinery to act as promising apoptosis-inducing agents, bearing high hopes for the management of cancers resistant to conventional treatments. [94]. This therapeutics can be used either alone or in combination with some of the conventional therapies. Several review articles have shed light to the great potential of apoptosis-targeted therapies [95, 96]. Some of which focus on Bcl-2 family proteins [97–99], IAPs [100], or c-FLIP [101] and the approaches that have been used to modify their activity to reactivate apoptosis and thus eradicate cancer cells.

As below, we refer readers to these reviews for specific details regarding the benefits of some novel therapeutic agents directed against some antiapoptotic targets, which have been shown to demonstrate enhanced apoptotic killing and sensitize resistant cancer cells to antineoplastic agents. Nevertheless, we show below a few of the most promising therapeutic strategies which target the induction of apoptosis.

### 3.1. Targeting Antiapoptotic Bcl-2 Family Members

The complex interplay between proapoptotic and antiapoptotic members of the Bcl-2 family plays a crucial role in cellular fate determination. Attempts to overcome the cytoprotective effects of Bcl-2 and Bcl-xL in cancer include three strategies: (1) shutting off gene transcription, (2) inducing mRNA degradation with antisense oligonucleotides, and (3) directly attacking the proteins with small-molecule drugs. Herein, we will provide some of the most promising strategies for modulating the activity of apoptosis genes and their proteins for cancer therapy.

Some members of the steroid/retinoid superfamily of ligand-activated transcription factors (SRTFs) represent potentially “drugable” modulators of Bcl-2 and Bcl-xL gene transcription although they are not components of the “core” apoptosis machinery. For example, expression of Bcl-2 is estrogen-dependent in the mammary gland. Consequently, antiestrogens, such as tamoxifen, inhibit endogenous Bcl-2 expression in breast cancer cell lines, promoting sensitivity to cytotoxic anticancer drugs such as doxorubicin. In addition to antiestrogens in estrogen receptor- (ER-) positive breast cancers, expression of Bcl-2 or Bcl-xL can be downregulated in specific types of cancer and leukemia cells by small molecule drugs that modulate the activity of retinoic acid receptors (RAR), retinoid X receptors (RXR), PPAR, vitamin D receptors (VDR), and certain other members of the SRTF superfamily. RAR and RXR ligands are already approved for treatment of some types of leukemia and lymphoma and are in advanced clinical testing for solid tumors. PPAR modulators have demonstrated antitumor activity in xenograft models of breast and prostate cancer [10], sometimes displaying synergy with retinoids, probably due, in part, to the fact that PPAR binds DNA as a heterodimer with RXR. Moreover, troglitazone, a potent PPAR agonist, can lower serum PSA in men with advanced prostate cancer; however, its proapoptotic features are not confirmed* in vivo* yet.

Compounds that inhibit histone deactylases (HDACs), called HDAC inhibitors, act as transcriptional repressors by interacting with retinoid receptors and other transcription factors. These inhibitors can modulate expression of Bcl-2 or Bcl-xL in some tumor lines [51]. These observations portend opportunities for exploiting endogenous transcriptional pathways for suppressing expression of antiapoptotic Bcl-2-family genes in cancer, together with the idea of employing them as chemo- or radiosensitizers, rather than relying on their antitumor activity as single agents. The genetic characteristics of cancer cells that dictate response or resistance to SRTF-ligands, as well as the complex pharmacological interplay between this class of agents and conventional cytotoxic drugs, need to be investigated more.

Because Bcl-2 antisense enhances sensitivity to cytotoxic anticancer drugs* in vitro* and in xenograft models, most clinical trials combine the antisense agent with conventional chemotherapy. More precisely, antisense oligonucleotides targeting the Bcl-2 mRNA have been introduced to Phase III clinical trials for melanoma, myeloma, CLL, and AML and Phase II activity underway for a variety of solid tumors. [102]. Moreover, Phase II data suggest a benefit from adding Bcl-2 antisense to conventional therapy, but definitive proof awaits the Phase III results.

Beside the antisense oligodeoxynucleutides (e.g., G3139 [103]), various drugs molecules that target Bcl-2 and Mcl-1 have been tested for their abilities to induce apoptosis in cancer cells [104]. Understanding how cells keep these antiapoptotic proteins controlled is the base on which the therapeutic potency for targeting the Bcl-2 and Bcl-xL proteins by these molecules is established. In this regard, a large family of endogenous antagonists of Bcl-2 and Bcl-xL has been revealed (so-called “BH3-only proteins”), possessing a conserved BH3 domain that binds a hydrophobic crevice on the surface of Bcl-2 and Bcl-xL [100]. Synthetic BH3 peptides generated as small-molecule drugs that occupy the BH3 binding site on Bcl-2 or Bcl-xL, abrogating their cytoprotective functions, have been validated [105]. Many research groups have presented preclinical data regarding BH3-mimicking compounds. The optimal structure-activity relation (SAR) profile of these compounds had been determined. These molecules showed broad-spectrum activity against the various antiapoptotic members of the Bcl-2-family (Bcl-2, Bcl-xL, Mcl-1, Bcl-W, Bfl-1, and Bcl-B), in terms of balancing antitumor efficacy. Of these molecules, which target Bcl-2, are the small molecule Bcl-2 inhibitors (e.g., HA14-1; [103]) and BH3 peptidomimetics [106]. The most prominent molecules among them are the Bcl-2 antagonists ABT-737 and ABT-263 [107, 108]. That novel Bcl-2/Bcl-xL/Bcl-W inhibitor (ABT-737) has been developed. It showed enhanced activity of chemotherapeutic agents or ionizing radiation in the preclinical studies. That compound displays impressive antitumor activity in human tumors including follicular lymphoma, chronic lymphocytic leukemia, and small cell lung cancer (SCLC)* in vitro* and* in vivo* [107] and in nonsmall lung cancer (NSCLC) [109].

ABT specifically bind to Bcl-2, Bcl-xL, and Bcl-W flipping them from Bak and Bax. ABT-737 mimics the BH3-only protein, Bad, by docking to the hydrophobic groove of antiapoptotic proteins, thereby disabling their capacity to antagonize the actions of proapoptotic proteins. Therefore, ABT-737 is highly potent (i.e., at nanomolar concentrations) in killing tumor cells which are dependent upon Bcl-2 for survival [110]. Although ABT targets almost all the proapoptotic family members of Bcl-2 except Mcl-1, it has been found that its combination with deoxyglucose has efficiently eliminated cancer cells* in vitro* and* in vivo* [111]. ABT-737 was modified at three sites to create improved ABT-263 for oral bioavailability without the loss of affinity to the Bcl-2 family of proteins [108]. As a single agent, however, ABT-263/737 (ABT) induces apoptosis only in limited tumor types, such as lymphomas and some small cell lung carcinomas [107, 108, 112].

Other strategies for countering Bcl-2 and Bcl-xL in cancer include over-expression of opposing proapoptotic family members such as Bax with p53 adenovirus (in Phase III trials) or with Mda7 (IL-24) adenovirus gene therapy (completed Phase I trials), as well as Bax adenovirus gene therapy for regional cancer control. Alternatively, it might be possible to activate the Bax and Bak proteins using drugs that mimic agonistic BH3 peptides [105].

One further strategy to counteract Bcl-2 family members is the monoclonal antibodies which target the tetra-span membrane protein CD20 (Rituximab) but can also downregulate expression of Bcl-2 family members, Mcl-1 (intrinsic pathway) and XIAP (convergence pathway) in certain leukemias, providing yet another example of unexpected links to apoptosis pathways through receptor-mediated signaling [113].

### 3.2. Targeting Cell Cycle Control System for Apoptosis Induction

The relationship between cell cycle arrest and apoptosis is complex. Signaling pathways following apoptosis-inducing stimuli either arrest the cell cycle following damage signals to allow time for repair or switch to initiation of apoptosis after apoptogenic agents. These agents, such as ionizing radiation or some chemotherapy, induce apoptosis in many cell types [114]. Apoptosis is frequently associated with proliferating cells. This implies the existence of molecules in late G1 and S phase, whose activities facilitate execution of the apoptotic process. Once the cells are committed to cell death, apoptogenic factors, including cytochrome* c*, are released from mitochondria to initiate a caspase cascade [115].

An important cell cycle regulator plays a central role in the regulation of cell cycle arrest and cell death is the tumor suppressor, p53 [116]. It has recently been discovered that the p53 activates apoptosis through parallel pathways that may depend on transcription events or not [117]. Under many types of stress, p53 induces cell cycle arrest and apoptosis to maintain genomic integrity and prevent damaged DNA being passed on to daughter cells. Tumor cells have inactivated p53. About 50% of this inactivation is achieved through mutations in its sequence and the rest by disabling key components that lie upstream or downstream of p53 in a common signaling pathway [118]. In p53 wild-type tumors, p53 may be compromised, by inactivation of positive regulators of p53 activity (such as p14ARF [119]) or over-activation of negative regulators of p53 activity (such as Akt [120]).

Bax is one of the best known downstream p53 transcriptional targets that directly affect apoptosis. A further transcription-independent role of p53 in apoptosis has been attributed to its ability to block the antiapoptotic function of Bcl-2 and Bcl-xL on the mitochondria [121, 122]. p53 promotes, directly or indirectly, the apoptotic activities of proapoptotic members of the Bcl-2 family, Bax and Bak [121, 123]. Moreover, after targeting DNA by some damaging agents, p53 contribute as a transcription factor. p53 transcriptionally upregulates genes such as those encoding p21WAF-1/CIP-1 and GADD45, which induce cell cycle arrest in response to DNA damage [124, 125]. However, p53 can trigger elimination of the damaged cells by promoting apoptosis through the upregulation of proapoptotic genes such as Bax, NOXA, TRAIL-R2 (DR5), and Fas (CD95/Apo-1) [12, 55, 126, 127]. However, the cell can choose between p53-dependent cell cycle arrest or apoptosis. How cells choose between this p53-mediated cell cycle arrest and apoptosis has three possible models. (I) One model suggests that more profound DNA damage induces higher and prolonged activation of p53, which increases the chances of apoptosis over arrest [128]. (II) Another model suggests that different cell types might keep different p53-regulated genes in regions of active chromatin, which determines the cassette of genes that are transcriptionally upregulated [129]. (III) A third model proposes that the availability of transcriptional cofactors determines the ability of p53 to activate different subsets of genes [130, 131].

DNA damage-inducing apoptotic factors induce the activation of upstream kinases such as ATM (ataxia-telangiectasia mutated), ATR (ATM and Rad-3 related), and DNA-PK (DNA-dependent protein kinase), which can directly or indirectly activate p53. Phosphorylation of p53 by upstream kinases inhibits its negative regulation by MDM-2, which targets p53 for ubiquitin-mediated degradation [132]. In fact, lack of functional p53 contributes to apoptosis resistance due to the inability to undergo p53-mediated apoptosis sometimes due to p53 mutations.* In vitro* studies have reported that loss of p53 function reduces apoptosis by 5-FU [57]. Other clinical studies have found that p53 overexpression (a surrogate marker for p53 mutation) correlates with resistance to apoptosis by 5-FU [133, 134]. Other studies have found no such correlation [135]. Such conflicting findings may be due, at least in part, to the fact that p53 overexpression does not actually reflect p53 mutation in as many as 30–40% of cases [136]. A recent study has suggested that certain p53 mutants may increase dUTPase expression, inhibiting apoptosis by 5-FU [137].

A number of* in vitro* studies have demonstrated decreased cisplatin-induced apoptosis in p53 mutant tumor cells [138–140]. Some studies have reported that disruption of p53 function actually enhances apoptosis by cisplatin [141, 142]. This enhanced apoptosis was attributed to defects in p53-mediated cell cycle arrest, which reduced time for DNA repair. Some tumors with mutant p53 have a worse clinical outcome which means failure to induce apoptosis by therapeutic drugs [143].* In vitro* data from other laboratories and others suggest that development of resistance to apoptosis by taxan is feasible in p53 null cells [144]. The clinical relevance of p53 status for taxan-induced is yet to be determined.* In vitro* studies have found that p53 status does not affect paclitaxel-induced apoptosis, [145–147]. On the other hand, doxorubicin was more active against p53 wild-type tumor xenografts than p53 mutant and null cells [148]. Furthermore, apoptosis induction by doxorubicin in acute lymphoblastic leukaemia cell lines was found to be dependent on the presence of wild-type p53 [149]. In the clinical setting, p53 mutations have been correlated with lack of response to doxorubicin in patients with locally advanced breast cancer [150]. These data indicate that doxorubicin is more active against p53 wild-type tumors. Fichtner et al. found no correlation between p53 status and sensitivity to the apoptogenic carboplatin, in xenotransplanted colorectal tumors [151]. Similarly, Jacob et al. found that p53 status did not correlate with CPT-11-induced apoptosis in a panel of colorectal cancer cell lines [152, 153]. Some studies have found that carboplatin induces apoptosis to a similar extent in isogenic p53 wild-type and null cancer cells [118]. In general, all the above mentioned studies suggest that p53 mutant tumors may be equally responsive to apoptosis inducers or possibly more sensitive than p53 wild-type tumors. That led to application of combinatorial drug therapy of paclitaxel and cisplatin for maximum apoptosis induction in p53 mutant ovarian tumors than p53 wild-type tumors as introduced [154].

#### 3.2.1. Cyclines

Another important family, critically controlling cell cycle, is cyclines [155, 156]. Here, we will focus on an important member of this family, cyclin E, which has direct relation with apoptosis signals. Cyclin E has been shown to have a Cdk2-independent function in regulating apoptosis of hematopoietic cells [157, 158]. The larger N-terminal truncation of cyclin E that generates p18-cyclin E prevents its binding to either Cdk2 or CKIs p21Waf1 or p27Kip1. Therefore, unlike the other isoforms of* cyclin E*, p18-cyclin E cannot bind Cdk2 and therefore interferes with Cdk2-dependent (bound to cyclin E1, E2, or A) kinase activity. Cleavage of cyclin E results in loss of its Cdk2 associated kinase activity and consequently its function in the cell cycle [157]. Recently, it has been reported that p18-cyclin E mediates p53 function-independent apoptosis by regulating the relationship between Bax and Ku70 [159]. That study's findings established a role for Ku70 in regulating Bax-mediated apoptosis in hematopoietic cells that generate p18-cyclin E. By interacting with Ku70, p18-cyclin E releases Bax from Ku70, thus allowing Bax to be activated during gentoxic stress and thereby leading to apoptosis [159]. Therefore, p18-cyclin E, Bax, and Ku70 emerge as key regulators of the apoptotic pathway at least in hematopoietic cells. The sensitivity of these cells to genotoxic stress can be explained by their ability to generate p18-cyclin E.

The cleavage of cyclin E can be prevented by Bcl-2 overexpression, indicating that Bcl-2 functions upstream of the mitochondrial apoptotic cascade [115, 158]. How Bax is released from its complex with Ku70 is still unknown. One mechanism may consist of a structural change in conformation of the Bax binding-domain of Ku70 upon binding of p18-cyclin E at the amino terminus. Another possibility might be the recruitment of histone acetyl transferases, which would acetylate several lysine residues at the carboxy terminus of Ku70 [160]. However, it is quite possible that other pathways and various feedback loops exist to activate Bax and thereby to amplify the apoptotic cascade in hematopoietic and other cell types.

It is now clear that, through its dual role, cyclin E provides a physiological balance between cell proliferation and death of hematopoietic cells [161]. Cyclin E has an initial limited activation of caspase-3 perhaps through a small amount of primed/activated mitochondrial Bax. Then, cyclin E is proteolytically cleaved by caspase-3 to generate p18-cyclin E, which interacts with Ku70 resulting in release of Bax from the Ku70-Bax complex. This contributes to a robust activation of Bax, leading to its mitochondrial targeting and amplification of the intrinsic pathway of apoptosis. This is consistent with the idea that limited caspase activation is not sufficient to release enough cytochrome c leading to significant apoptosis, at least, in hematopoietic cells. Rather, an amplification loop is required to trigger massive cytochrome c release from mitochondria resulting in abundant caspase-3 activation and cell death [115]. Caspase-3 and caspase-7 may participate in a feedback amplification loop to promote the mitochondrial apoptotic pathway [162].

#### 3.2.2. Ku70, from Cyclin E to Bax

As we previously mentioned, the key regulatory step in the intrinsic cell death pathway is the activation of the proapoptotic molecule, Bax [163]. Although the mechanism of Bax activation remains unclear, a recent study indicates that Bax is kept inactive in some cells, to counteract apoptosis, by interacting with cytosolic Ku70 [163, 164]. Overexpression of Ku70 prevents Bax-mediated apoptosis, whereas targeting Ku70 causes cells to become more sensitive to a variety of apoptotic stimuli. Importantly, we showed that some of these apoptotic stimuli which are not directly targeting DNA break like the microtubule stabilizing agents, Taxane, and hyperthermia stimulated caspase-dependent apoptosis after Ku70 inhibition (unpublished data). These results demonstrated that Ku70 is a physiological inhibitor of Bax-induced apoptosis; a finding that expands on Ku70's previously known role in DNA repair [163], particularly through nonhomologous end joining (NHEJ). Moreover, cells from Ku70 knockout mice are hypersensitive to agents that induce apoptosis in the absence of DNA damage, such as staurosporine [159]. This suggests that Ku70 plays a role in suppressing apoptosis independently of its role in DNA repair [165]. Based on these findings, nuclear Ku70 is therefore considered to be mainly responsible for repair of DNA damage, whereas the cytosolic pool of Ku70 may be primarily a regulator of Bax activation [162, 164]. Therefore, Ku70 plays a dual role in NHEJ and regulation of Bax, which in turn may determine the balance between cell survival and programmed cell death in hematopoietic cells. Ku70 may not be unique in assuring Bax sequestration in the cytosol. Other Bax interactive proteins such as the peptide humanin [166], the apoptosis repressor with caspase recruitment domain (ARC) [167], or crystalline [168] may also function in various cellular systems to sequester Bax. On the other hand, after apoptotic stimulation other Bax-interacting proteins, such as p53 [169] and Bif- [170] and apoptosis-associated speck-like protein (ASC) [171], and MOAP-1 [172] promote Bax conformational change and mitochondrial translocation.

#### 3.2.3. Nonapoptotic Function of Caspases

Although caspases are classically known for their role in apoptosis, their involvement in biological processes apart from cell death has recently received increased attention. For example, they play an important role in the inflammatory signaling pathways [173, 174]. The nonapoptotic functions of these proteases suggest that they may become activated independently of the apoptotic cascade, thus leading to the cleavage of specific substrates, such as kinases, cytokines, transcription factors, and polymerases.

Functional analysis of conditional caspase-deficient mice or derived cells confirmed the crucial roles of caspases in cell proliferation, differentiation, and inflammation. It has been reported recently that caspase-3 is a negative regulator of B-cell cycling. This study shows that while the apoptotic pathway is largely unaffected in caspase-3 knockout mice, splenic B-cell proliferation is enhanced* in vivo*, and in response to mitogenic stimulation* in vitro*, hyperproliferation is seen. Genetic and biochemical data demonstrate that caspase-3 is essential for the regulation of B-cell homeostasis [175]. In contrast to caspase-3, caspase-8 is a positive regulator of cell cycling as B-cell proliferation since caspase-8 deficient mice fail to proliferate [176, 177]. Recently, it has been suggested that caspase-3 and caspase-7 together play a role in development, since double knockout mice exhibit defects in heart development, leading to death immediately after birth. In contrast, knockout of either caspase individually on the same genetic background resulted in viable animals.

### 3.3. Targeting DNA Repair System for Apoptosis Induction

DNA repair can determine fate of a cell with or without treatment stress which either resists over to survive or respond to toxic agents. When the repair mechanisms are unsuccessful, it may cause cellular senescence (permanent cell cycle arrest), oncogenesis, or apoptosis which plays an essential role in survival of the organisms by preventing the multiplication of mutated chromosomes, as well as elimination of indisposed cells, normal embryonic development, and maintenance of cell homeostasis. [178]. In cancer treatments, apoptosis-inducing chemotherapeutic drugs induce DNA damage either directly (e.g., platinum drugs) or indirectly (e.g., 5-FU and topoisomerase poisons). The response to DNA damage is either repair or cell death. Only when repair is incomplete, for example, when the DNA damage is too extensive, cells will undergo apoptosis. Herein, we describe some major mechanisms through which cells can overcome apoptosis by damaging agents and we introduce some example molecules which had successfully targeted in some types of cancer to stimulate or enhance apoptosis by therapeutic agents.

Nucleotide excision repair (NER) is the major pathway for DNA repair after DNA stress. However, for example, cisplatin induces platinum-DNA adduct which could be removed by NER as challenge mechanism by cancer cell to repair of platinum-induced DNA damage [178]. Defects in NER result in hypersensitivity to cisplatin, and that restoration of NER activity reduces sensitivity to more normal levels [179]. NER is a complex process involving at least 17 different proteins; however, upregulation of only a few rate limiting components of the NER system is necessary to increase a cell's capacity for NER [180]. One of these important rate-limiting factors is the excision repair cross-complementing 1 protein (ERCC1), which plays a crucial role in response to apoptosis inducer, cisplatin. Increased expression of ERCC1 associated with cisplatin resistance [181–183]. Clinically, high levels of ERCC1 are correlated with poor response to platinum-based chemotherapy in ovarian, gastric, and nonsmall cell lung cancers (NSCLC) [184–186]. In addition, high mRNA expression of ERCC1 and thymidin synthase (TS) has been acting as predictors for poor response to combined oxaliplatin/5-FU treatment of advanced colorectal cancer [187]. Targeting ERCC1 expression, using an antisense expression construct, made ovarian cancer more sensitive to cisplatin than controls in cell line and xenograft models [188]. Another central component of the NER machinery, xeroderma pigmentosum group A (XPA), has been found to be overexpressed in apoptosis resistant cancer cells under apoptosis inducer, cisplatin, treatment [184]. Collectively, these studies suggest an important role for NER in mediating resistance to DNA damage and subsequent apoptosis by platinum.

Another DNA damaging agent is 5-FU. 5-FU treatment induces TS inhibition which subsequently causes nucleotide imbalances that severely disrupt DNA synthesis and repair [189]. TS inhibition results in the accumulation of deoxyuridine triphosphate (dUTP), as the essential conversion process of deoxyuridine monophosphate (dUMP) to deoxythymidine monophosphate (dTMP) is blocked [190]. Both dUTP and another 5-FU metabolite, fluorodeoxyuridine triphosphate (FdUTP), can be misincorporated into DNA. Repair of uracil and 5-FU-containing DNA could be achieved by the base excision repair enzyme uracil-DNA-glycosylase (UDG) [191]. However, this repair mechanism is futile in the presence of high (F)dUTP/dTTP ratios causing false nucleotide incorporation. These futile cycles of misincorporation, excision, and repair eventually lead to DNA strand breaks. However, some cells show resistance to this mechanism by increased dUTPase. The increased dUTPase expression has been associated with resistance to TS inhibitors like 5-FU [192–194].

Another mechanism is the DNA mismatch repair (MMR) which is an important mechanism that controls the decision from survival to apoptosis. The main function of the MMR system is to scan newly synthesized DNA and remove single nucleotide mismatches that arise during replication. MMR deficiency is implicated in the development of apoptosis-resistance against wide range of DNA-damaging agents, including platinum drugs [195]. It is possible that MMR recognition of DNA damage may trigger an apoptotic pathway or that futile cycles of DNA damage/repair mediated by the mismatch repair machinery generate lethal DNA strand breaks [196]. MMR has a role beyond that of repair in response to DNA damage. Inherited defects in the DNA MMR genes, especially hMLH1 and hMSH2, are common in certain familial forms of cancer such as hereditary nonpolyposis colon cancer (HNPCC). Such defects were also observed in a variety of sporadic tumors, including colorectal, breast, and ovarian cancers [197–200]. DNA MMR deficiency gives rise to the microsatellite instability (MSI) phenotype, which is detected as variations in lengths of DNA repeat sequences present in the genome [201]. Cisplatin-induced apoptosis and acquisition of the drug resistance were found to be associated with hypermethylation of the hMLH1 promoter [202]. One clinical study found that ovarian tumors that were initially microsatellite stable before cisplatin-based stress exhibited MSI in the residual tumors after chemotherapy, and that was proposed to be due to loss of hMLH1 expression [203]. Hence, preclinical studies strongly implicate loss of MMR, in particular loss of hMLH1, in overcoming apoptosis by cisplatin. Reversal of hMLH1 promoter methylation by DNA methyl transferase inhibitor, 2-deoxy-5-azacytidine (DAC), has been shown to resensitize cells to a range of apoptotic agents, including platinum drugs [202]. Thus, DAC has now entered clinical trials in combination with carboplatin in some cancers. Finally, a clinical study found that MMR deficiency was a predictive factor for apoptosis induction by carboplatin in advanced colorectal cancer [204]; however, MMR deficiency had no effect on sensitivity to the non-DNA-targeted apoptosis-inducing agents, paclitaxel and docetaxel.

In addition to the above mentioned repair mechanisms and other several repair machineries, such as mutagenic repair, which may become effective for the recovery of genome against constant attack of numerous genotoxins, UV-radiation, ionizing radiation, and various chemicals are responsible for most of the mutagenesis due to a process of translesion that inserts an incorrect nucleotide opposite to the lesion and then continues elongation [205]. Targeting any of such mechanisms could enhance apoptosis instead of the repair and eradicate the defectively repaired cells under apoptotic inducers.

#### 3.3.1. DNA Double Strand Break Repair and Apoptosis

Double-strand breaks (DSBs) repair mechanism is one of the widespread mechanisms which efficiently repairs double-strand breaks and single-strand gaps in damaged DNA by a series of complex biochemical reactions, as a result of ionizing radiation, UVR, ROS, and chemotherapeutic genotoxic chemicals [205]. The lethal effects of double strand breaks (DSBs) can be conquered by the existence of two independent pathways, such as homologous recombination (HR) and nonhomologous end joining (NHEJ). Multiple proteins are required for DSB repair by recombination, which are conserved among all eukaryotes. Deficiencies in such repair mechanism can develop cancer.

#### 3.3.2. BRCA1

BRCA1 is a tumor suppressor gene that regulates cellular responses to DNA stress by apoptotic inducers. Germline mutations of the BRCA1 gene account for about 10% of breast and ovarian cancer cases, and lower than normal BRCA1 expression may be an important factor that contributes into sporadic cancers [206, 207]. Recently, BRCA1 has been found to reside in a large DNA repair complex that includes various mismatch repair proteins including hMLH1 and hMSH2; thus, it plays a role in DNA repair [208]. BRCA1 also plays a role in the activation of cell cycle checkpoints in response to different cellular stresses including DNA damage and disruption of microtubule dynamics [209, 210]. Now, BRCA1 has been implicated in the regulation of apoptosis [211]. It appears that, similar to p53, BRCA1 may function as a sensor of cell stress by relaying signals to either the cell-cycle checkpoint machinery or cell death machinery. A recent study by Quinn et al. found that BRCA1 acts as a differential modulator of chemotherapy-induced apoptosis in breast cancer cells [212]. They found that BRCA1 enhanced sensitivity to apoptosis induced by antimicrotubule agents, such as paclitaxel and vinorelbine, but inhibited apoptosis induced by DNA-damaging agents such as cisplatin and etoposide. Moreover, inhibitors of poly (adenosine diphosphate- (ADP-) ribose) polymerase (PARP) show the synthetically lethal effect in BRCA1-defective tumors because BRCA1 encodes protein that is required for efficient homologous recombination (HR) [213].

#### 3.3.3. Ku Protein, from Gatekeeping to Caretaking

Double strand break (DSB) repair includes homologous recombination (HR) and nonhomologous end joining (NHEJ). DSB repair through HR process is an error free pathway, since it requires an extensive region of sequence homology between the damaged and template strands, whereas NHEJ is an error prone alternate pathway for the repair of DSBs, which essentially joins broken chromosomal ends independent of sequence homology. The NHEJ process is initiated by the binding of specific protein to the broken ends, which may act as end bridging factor [214]. The catalytic subunit of DNA protein kinase (DNA-PKcs) is required in mammalian NHEJ to bridge the DNA ends through their protein-protein interactions [215].

Cancer susceptibility genes have been categorized into two classes, namely, caretakers and gatekeepers. Caretakers are involved in DNA repair and whose inactivation can lead to genomic instability while gatekeepers control cell death and proliferation. Loss of functions in both caretaker and gatekeeper genes results in an increase in cancer susceptibility. Ku86 and p53 are examples of such caretaker and gatekeeper, respectfully. Their functions are closely linked [216]. Ku is a caretaker gene that maintains the integrity of the genome by a mechanism that suppresses chromosomal rearrangements. Ku complex (a heterodimer of Ku70/Ku80 [*≈*86]) is a major end binding factor in mammalian cells, possessing end bridging activity [217, 218]. Ku exists as a heterodimeric DNA binding complex in eukaryotes, consisting of two protein subunits of about 70- and 80-kDa, known as Ku70 and Ku80 (in* S. cerevisiae*) or Ku86 (in higher eukaryotes). This complex was originally identified two decades ago as a major target of autoantibodies from Japanese patients with scleroderma-polymyositis overlap syndrome [219]. Functional Ku proteins are critical for the maintenance of genomic stability, DNA repair, and hence cellular and organismal viability [220]. Li and colleagues reported the putative tumor suppressor function of Ku70. On the other hand, Ku was identified as a nuclear protein involved in both homologous recombination (HR) or nonhomologous end joining (NHEJ). Moreover, Ku proteins have been implicated in numerous other cellular processes, including telomere maintenance, antigen receptor gene arrangements (e.g., variable (diversity) joining {V(D)J} recombination), regulation of specific gene transcription and apoptosis, regulation of heat shock-induced responses, and a newly identified role in regulation of the G2 and M phases of the cell cycle [221]. Moreover, an association of the DNA-PK-Ku70-Ku86v with a number of cell cycle regulatory proteins such as p53, CDK4, and E2F-4 had been reported, suggesting a pivotal role of Ku in cell cycle regulation and malignant transformation [222].

Recently, Ku70 has been shown to bind to the proapoptotic protein BAX and inhibit BAX-mediated apoptosis* in vitro* by preventing its relocalization to the mitochondria [223]. This antiapoptotic function is mediated by a domain in the carboxy-terminal of Ku70 and does not require the cooperative effects of Ku80. Although the exact function of Ku in these processes is presently still not clear, what is certain is that this protein is of fundamental importance in cell viability especially under treatment stress [223]. Hence, the idea of targeting Ku70 had emerged to enhance apoptosis by different therapies. That was because tumor cells depend on DNA repair mechanisms to a greater extent than normal cells; hence, many cancer therapies target such DNA repair machinery [224]. As DNA-PK plays a crucial role in the DSBR, the kinase activity of the DNA-PK complex is regulated through the DNA end-binding (DEB) activity of its regulatory subunit Ku. Therefore, the regulation of Ku expression and function also plays a vital role in cancer cells resistance to anticancer therapy. Thus, targeting Ku protein led to changes in susceptibility to anticancer drug-induced apoptosis [225, 226]. Most exciting are the new clinical studies that target Ku as their primary strategy. Reports have shown that the status of Ku or NHEJ in tumors can enhance apoptosis by radiotherapy or chemotherapy, suggesting that Ku may be a potential target to overcome resistance during cancer treatment. Recently, novel therapies such as the engineering of selective small molecule, DNA-PK inhibitors, that enhance radiation-induced tumor control in a mouse-human xenograft model of cancer have been developed and have shown promising results [224]. Other examples include the use of adenovirus-mediated, heat activated antisense Ku70 expression that radiosensitizes human tumors [227] and the use of a Ku antibody to block MM cell adhesion and abrogates the protective effect of membrane Ku [228].

Further understanding of the possible link of the main functions of Ku in different cell systems may also help in answering the intriguing question of how autoantibodies against Ku are generated in various autoimmune diseases. This provides an exciting insight into the future of anticancer development. It has shown that Ku70 siRNA sensitized mammalian cells to radiation and topoisomerase II inhibitor, etoposide [229]. Recently, small molecule, HDAC inhibitors, which targets Ku70 acetylation enhanced DNA damage by DNA-damaging agents in prostate cancer and they enhanced radiation effect in melanoma cells [230, 231]. Moreover, Subramanian used HDAC inhibitors, which target ku70 acetylation to induce apoptosis in neuroblastoma cells [163]. These molecules increase the acetylation of Ku70 in the cytoplasm, resulting in the release of Bax from Ku70. Subsequently, activated Bax translocates to the mitochondria. In our laboratory we identified Ku70, particularly as a required molecule for the cytostatic arrest under hyperthermia treatment in nonsmall lung cancer cells. In that study, small interference RNA against Ku70 could inhibit the cytostatic arrest and switch cells to cytotoxic arrest and caspase-dependent apoptosis mediated by Bax activation [232].

### 3.4. Targeting Death Receptors (DR)

Many tumors refract to the classic apoptosis-inducing cancer therapies which provoke intrinsic pathway-based apoptosis due to development of defects in that pathway under treatment stress [233]. To enhance cancer cell apoptosis and thus overcome treatment failure, many therapeutic strategies targeting other molecules implicated in apoptosis resistance have been developed [95, 96]. Hence, alternative therapies which provoke the extrinsic pathway-based apoptosis were developed. For example, attempts to apply TNF as a cancer treatment were stymied by the proinflammatory effects of this cytokine, because it induces both caspase activation pathways and NFKappaB. Fortunately, the TNF family cytokines, FasL and TRAIL, trigger caspase activation without concomitant induction of NFKappaB giving chances for successful cancer therapy via apoptosis, where TNF failed due to toxicity. The antibodies that trigger the receptor Fas (CD95) unfortunately showed high toxicity to liver [224], while TRAIL and agonistic antibodies that bind TRAIL receptors appear to be well tolerated* in vivo*. As a fact, Phase I trial in humans was recently completed using an agonistic antibody directed against TRAIL-receptor-1 (TRAIL-R1; DR4). In mouse xenograft models bearing human tumor cells lines, TRAIL and its agonistic antibodies directed against TRAIL receptors have been demonstrated to possess potent antitumor activity [234], supporting the idea of using these biological agents as a novel approach to cancer treatment and thereby mimicking some of the effector mechanisms normally employed by the immune system in its defense against transformed cells and potentially bypass the defective intrinsic (mitochondrial) pathway to apoptosis.

Synthetic triterpenoids, such as CDDO and CDDOm, sensitize solid tumor cell lines to TRAIL and induce apoptosis as single agents in leukemia cells, through a caspase-8-dependent mechanism that remains operative even in chemorefractory cells [235–237]. Moreover, in leukemia, the protein kinase C (PKC) modulator byrostatin induces myeloid leukemia cell lines to produce TNF, resulting in autocrine engagement of TNF-receptors and apoptosis induction through a mechanism that is suppressible by TNFR-Fc fusion protein and caspase-8 dominant-negative [238]. Similarly, all-trans-retinoic acid (ATRA) induces TRAIL production and triggers autocrine induction of apoptosis in acute promyelomonocytic leukemia (APML) cells that harbor the RAR-PML fusion protein resulting from t (15; 17) chromosomal translocations [239].

TRAIL, a candidate for targeted therapy, which can preferentially kill cancer cells, is frequently hampered by various mechanisms of cancer cell resistance to apoptosis [240, 241]. As a cytokine, TRAIL induces apoptosis by binding one of its cognate death receptors and plays an important role in immune surveillance against tumors [49, 240, 241]. Nevertheless, in many types of cancer cells, effective antitumor activity of TRAIL requires the suppression of aberrantly expressed negative regulators of apoptosis [240, 241]. In general, as multiple cell signaling mechanisms may control apoptosis, cancer cells can employ a number of different strategies to suppress a protective apoptotic response [6–8]. From other side, survival signaling pathways are linked to the apoptotic machinery. These pathways can modulate components of the apoptotic machinery itself or key regulatory molecules within the core apoptotic pathways [242, 243]. Notably, various upstream signaling pathways often impinge on the same few central apoptosis control points, which involve some crucial members of the Bcl-2 family, inhibitor of apoptosis (IAP) proteins, and FLICE-inhibitory protein (c-FLIP) [6, 7, 38, 40].

### 3.5. NF-*κ*B as a Target for Apoptosis Induction

NF-*κ*B is a transcription factor that was discovered in the nucleus of B cells and binds to the enhancer of the kappa light chain of immunoglobulin. It is expressed widely in the cytoplasm of all types of cells. NF-*κ*B is an important molecular link between chronic inflammation, cell cycle, cancer development, and cell death [6, 244–247]. The transactive NF-*κ*B suppresses apoptosis by inducing the expression of some apoptosis-inhibitory genes, including IAPs, cFLIP, TNF receptor associated factor 1 (TRAF1), and TRAF2 [248]. Two typical prosurvival NF-*κ*B targets are Bcl-xL and XIAP, which can block apoptosis at multiple steps [249, 250]. Importantly, Chuang et al. demonstrated that a wide range of cytotoxic drugs (5-FU, doxorubicin, paclitaxel, and cisplatin) activated NF-**κ**B in a panel of cancer cell lines [251]. This suggests that NF-**κ**B activation is a general feature of cancer cell response to chemotherapy. For instance, increased NF-**κ**B activity in patients with oesophageal cancer has been correlated with reduced response to neoadjuvant chemotherapy and radiotherapy [252]. Now it is believed that NF-**κ**B appears to be a critical determinant of drug resistance; its activation reduces apoptosis by chemotherapy [247]. A number of* in vitro* studies demonstrated that inhibition of NF-**κ**B sensitizes cancer cells to chemotherapy-induced apoptosis [253–255]. Furthermore, NF-**κ**B is believed to be a major target for proteasome inhibitors, as proteasome inhibition prevents degradation of I**κ**B, blocking NF-**κ**B nuclear translocation [255, 256]. Clinical trials with proteasome inhibitors such as bortezomib are underway to inhibit NF-**κ**B signalling and enhance drug-induced apoptosis in cancers.

### 3.6. Targeting Multiple Pathways Regulators

Like antiapoptotic Bcl-2 proteins overexpression, IAPs overexpression is associated with poor prognosis and chemoresistance in many cancers [257–259]. It acted as a therapeutic target for apoptosis-inducing strategies [260]. Antisense oligonucleotides against XIAP and survivin have been developed [249]. In addition small-molecule inhibitors that bind to the BIR2 or BIR3 domain of XIAP, cIAP1, and cIAP2 enhance apoptosis [249]. Most of small-molecule IAP antagonists are SMAC mimetics, several of which are in advanced preclinical or early clinical development. Bivalent SMAC mimetics, which bind to both the BIR2 and BIR3 domains within a single molecule of XIAP as well as the BIR3 domains of two cIAP molecules, induce their dimerization, and subsequently trigger their proteasome mediated degradation, are more significant potent than their monovalent counterparts [257, 258]. Despite evidence indicating that SMAC mimetics show great promise for cancer therapy [257], they can induce loss of cIAP1 and cIAP2, resulting in NIK stabilization and consequent NF-kB activation [48, 257].

Targeting c-FLIP appears to be a highly promising therapeutic strategy to reduce the apoptotic threshold because its overexpression can protect cancer cells from both TRAIL and chemotherapy-induced apoptosis, while small interfering RNA- (siRNA-) mediated downregulation of c-FLIP is able to sensitize cancer cells to FASL, TRAIL, and chemotherapeutic agents [39, 101]. Targeting FLIP by siRNAs in a variety of cancer cell types showed their potential as therapeutic agents to induce apoptosis [101]. Nevertheless, the widespread use of such strategy in clinical settings depends on the safety delivery of siRNA [261]. Thus, many research efforts have been devoted to improve RNA interference (RNAi) therapeutics, which lead to important advances in the field [262, 263]. In May 2008, the first Phase I clinical trial for the treatment of solid tumors involving systemic delivery of siRNA via targeted nanoparticles was initiated (ClinicalTrials.gov identifier: NCT00689065) [262]. Importantly, data from this trial demonstrated, for the first time, that systemically delivered siRNA can reduce protein levels of a specific gene through an RNAi mechanism in humans [264]. This finding opens the gate for future application of siRNA as a gene-specific tool for cancer treatment, clinically. These applications facilitate targeting the antiapoptotic genes' products to kill cancer cell either alone or in combination with classic therapies. Recently, c-FLIP and other antiapoptotic proteins are promising targets for the development of RNAi therapeutics [101]. As well as RNAi-mediated downregulation of c-FLIP, RNAi-based reduction of Bcl-2, Bcl-xL, XIAP, and survivin has also been shown to sensitize cancers cells to a range of cancer therapies, including chemotherapeutic drugs and TRAIL [265].

### 3.7. Targeting Heat Shock Chaperons

#### 3.7.1. HSP90

Heat shock proteins 90 (Hsp90s) are abundantly and ubiquitously expressed proteins required for the energy-driven stabilisation, conformation, and function of a large number of cellular proteins, named clinets [266, 267]. Several key Hsp90 proteins are involved in the processes characteristic to the malignant phenotype, such as invasion, angiogenesis metastasis, and treatment resistance [268–270]. They also contribute to leading mechanism of mitogen-activated protein kinases (MAPK) and nuclear factor kappa B (NF-*κ*B) induction [271–273]. Moreover, Hsp90 stabilises Raf-1, Akt, and ErbB2 proteins [274–276], which are known to be associated with protection against radiation-induced cell death [277–279]. Molecular studies suggested that inhibiting HSP90 by targeted therapy could provide a promising strategy to enhance apoptosis by conventional therapies [280–286]. The inhibitor of Hsp90, geldanamycin, and its derivatives successfully enhance the radiosensitivity of tumor cell lines derived from different origins, including glioma, prostate, pancreas, and cervix [276, 280–284, 287]. However, geldanamycins have several limitations, including poor solubility, formulation difficulties, hepatotoxicity, and extensive metabolism by polymorphic enzymes, along with drug efflux by P-glycoprotein; therefore, efforts to design small synthetic inhibitors of Hsp90 with improved bioavailability and lower toxicity are devoted [288–291]. Now, pyrazole resorcinol compounds act as stronger inhibitors of Hsp90 than geldanamycin derivatives. Currently, the isoxazole resorcinol NVP-AUY922 shows the highest affinity for the NH2-terminal nucleotide-binding site of Hsp90 [290, 291], whereas NVP-BEP800 represents a novel fully synthetic, orally available 2-aminothieno [2,3-d] pyrimidine class Hsp90 inhibitor [292]. Both compounds have good pharmaceutical and pharmacological properties. They also exhibit strong antiproliferative activity against various tumor cell lines and primary tumors* in vitro* and* in vivo* at well-tolerated doses [292]. The novel inhibitors of Hsp90 can sensitize various tumor cells to apoptosis by destabilisation and depletion of several Hsp90 client proteins, thus causing the depletion of S phase and G2/M arrest by heat shock, increased DNA damage, and repair protraction and finally apoptosis [293].

#### 3.7.2. Clusterin

Clusterin (CLU) is a cytoprotective heat chaperone protein, involved in numerous physiological processes important for carcinogenesis and tumor growth, including apoptotic cell death, cell cycle regulation, DNA repair, cell adhesion, and theromprotection [294]. It is now accepted that the primary function of the 67–80 kDa cytoplasmic CLU (sCLU) protein form is cytoprotective as a stress response gene. sCLU expression is consistently reported to be increased with many apoptosis-inducers, chemotherapy or radiotherapy, treatment as an adaptive cell survival molecule* in vivo* and* in vitro* to block apoptosis [295]. That was also shown in human tumor tissues from prostate [296, 297], kidney [298], breast [299], ovarian [300], colon [301], lung [302], pancreas [303], cervix [304], glioma [305], and anaplastic large cell lymphoma [306].

It has recently been shown that sCLU knockdown in human cancer cells, using siRNA-mediated CLU gene silencing, induces significant reduction of cellular growth and higher rates of spontaneous apoptosis [294]. Thus, we consider the fact that clusterin, as a chaperon molecule, has been found to bind with the active form of Bax under apoptotic stimuli inhibiting its dimerization in the mitochondria and block apoptosis. Consequently, it has been hypothesized that sCLU gene silencing using siRNA or other techniques may ultimately develop into attractive antitumor apoptotic induction [294]. Thus, many researchers targeted sCLU expression silencing using antisense oligonucleotides (ASO) or RNAi, as promising tools for cancer therapy [307–309]. However, that was more effective when given in combination with convention therapies to synergize the effect of such combination therapy [310–312]. The ASO was challenged by the rapid intracellular degeneration of oligonucleotides in* in vivo* experiments. That opened the gate for inventing the first generation ASO in which the phosphoryl oxygen of DNA was replaced with a sulphate to create a phosphothiate backbone, ASOs, intended for cancer therapy. Recently, more modifications were made to the ribose, the 20-position, to improve the pharmacokinetic characteristics of second-generation phosphothioate ASOs, for example, OGX-011 [313].

In advanced breast cancer, targeting CLU by OGX-011 enhanced the apoptotic effect by Trastuzumab, an HER-2-targeted monoclonal antibody used in the clinical management of advanced breast cancer patients. Importantly, only the combination of OGX-011 and Tratuzumab leads to activation of apoptosis that was not observed with either agent alone. Phase I and phase II studies have suggested a combined therapy using ASOs against both of CLU and Bcl-2, along with Trastuzumab for advanced breast cancer patients [314, 315]. Targeting CLU by ASO enhanced apoptosis by paclitaxel or radiation in PC-3, prostate cancer cells [314].

Phases I and II trials in prostate cancer have shown that OGX-011 significantly enhanced the apoptotic response and efficacy of chemotherapy, radiation, and androgen withdrawal by inhibiting the expression of CLU. In other prostate cancer phase I trials, OGX-011 was given prior to radical prostoctomy, while some “well tolerated” phase II trials were established based on the biologic effectiveness of OGX-011 [315].

In our laboratory we reported for the first time the association between upregulation of the sCLU and persistence against apoptosis by paclitaxel in ovarian cancer cells and human tumors. Importantly, when we targeted CLU either by OGX-011 or RNAi we successfully enhanced caspase-dependent apoptosis and the cells restored their sensitivity to paclitaxel [144]. Similarly, CLU ASO enhanced cisplatin-induced apoptosis, human bladder cancer cells, and human lung adenocarcinoma both* in vitro* and* in vivo* [304].
